# Long non-coding RNA 00960 promoted the aggressiveness of lung adenocarcinoma via the miR-124a/SphK1 axis

This article has been retracted.

**DOI:** 10.1080/21655979.2021.1996507

**Published:** 2022-01-09

**Authors:** Zhipeng Ge, Haibo Liu, Tao Ji, Qiaoling Liu, Lulu Zhang, Pengchong Zhu, Liang Li, Liangming Zhu

**Affiliations:** a Weifang Medical University, Weifang, People’s Republic of China; b Department of Thoracic Surgery, Jinan Central Hospital Affiliated to Shandong University, Jinan, Shandong Province, P.R. China; c Chest Endoscopy Minimally Invasive Area, Shandong Provincial Chest Hospital, Jinan, Shandong Province, China; d Research Center of Basic Medicine, Central Hospital Affiliated to Shandong First Medical University, Jinan, China; e Department of Orthopaedics, Jinan Central Hospital Affiliated to Shandong University, Jinan, Shandong, China; f Department of Thoracic Surgery, Shandong Provincial Hospital Affiliated to Shandong University, Jinan, Shandong, China

**Keywords:** LINC00960, lung adenocarcinoma, aggressiveness, SphK1, miR-124a

## Abstract

Long non-coding RNAs (lncRNAs) are closely associated with the development of lung adenocarcinoma (LADC). The present study focused on the role of LINC00960 in LADC. miRNA and mRNA expression levels were detected using quantitative reverse transcription-polymerase chain reaction (qRT-PCR). Cellular functions were evaluated by MTT, colony formation, and Transwell assays, respectively. LINC00960 Luciferase and RNA pull-down assays were performed to clarify the interaction between miR-124a and LINC00960 or Recombinant Sphingosine Kinase 1 (SphK1). We observed that LINC00960 was overexpressed in LADC tumor tissues and cell lines. LINC00960 knockdown suppressed the proliferation, migration, and invasion of LADC cells. Moreover, LINC00960 sponged miR-124a to inhibit the SphK1/S1P pathway in LADC cells. LINC00960 knockdown markedly reduced the rate of tumor growth. The luciferase reporter assay results demonstrated an interaction between miR-124a and LINC00960 or SphK1. This interaction was confirmed using the RNA pull-down assay. In addition, miR-124a downregulation or SphK1 upregulation reversed the inhibitory effects of LINC00960 knockdown on cellular functions of LADC cells, suggesting that LINC00960 may be a potential therapeutic biomarker for LADC via the miR-124a/SphK1 axis. Accordingly, LINC00960 may be a potential therapeutic biomarker for LADC.

## Introduction

Lung cancer is the most common cause of tumor-associated mortality worldwide [1]. Non-small cell lung cancer (NSCLC) accounts for 85–90% of all cases [2,3] and is typically classified into three categories: atypical adenomatous/adenocarcinoma *in situ*, minimally invasive adenocarcinoma, and invasive adenocarcinoma [4]. Lung adenocarcinoma (LADC), as a type of invasive adenocarcinoma is characterized by insidious disease onset and high infiltration rates [4,5]. Moreover, LADC reportedly results in hematogenous and lymphatic metastasis by promoting vascular and lymphatic invasion [6]. Patients with LADC often exhibit no clear respiratory symptoms at an early stage; however, the 5-year overall survival rate following surgical resection is less than 10% [7]. The major strategies for treating LADC include surgery, chemotherapy, radiotherapy, targeted therapy, and immunotherapy [8]. Although targeted therapy can partially improve the prognosis of patients with LADC, the ability of the disease to easily metastasize, drug resistance, and low response rates remain persistent challenges that need to be resolved [9]. Therefore, in-depth studies examining the molecular mechanisms underlying LADC are of great importance in the quest to identify effective therapeutic targets for LADC.

Long non-coding RNAs (lncRNAs) are a family of endogenous RNAs with >200 nucleotides [10–12]. In LADC, dysregulated lncRNAs function as anti-tumor genes or oncogenes. For instance, the overexpression of lncRNA DGCR5 exacerbates the progression of LADC and predicts poor outcomes [13]. Upregulated lncRNA TTN-AS1 contributes to the proliferation and epithelial-mesenchymal transition of LADC [14]. However, overexpression of GMDS-AS1 inhibits the aggressiveness of LADC cells [15]. LINC00960, a newly discovered lncRNA, functions as an oncogene in bladder cancer and pancreatic ductal adenocarcinoma [16,17]. Moreover, the dysregulation of LINC00960 has been associated with lung disorders, such as idiopathic pulmonary fibrosis [18]. However, the potential of LINC00960 in LADC remains unclear. MicroRNAs (miRNAs) are a group of small non-coding RNAs [19]. The aberrant expression of miRNAs predicts poor clinical results and aggressiveness of tumor cells, including NSCLC [20–23]. miR-124a was first identified in the central nervous system [24,25]. Downregulation of miR-124a is associated with the development of NSCLC. Accordingly, miR-124a is a novel diagnostic and prognostic chemotherapeutic biomarker for NSCLC [26,27]. However, the underlying mechanisms remain unclear.

Sphingosine kinases (SphKs) are rate-limiting enzymes that regulate sphingosine-1-phosphate (S1P) synthesis; SphK1 is an isozyme of SphK [28]. As a widely occurring secondary messenger molecule, S1P is a vital regulator of various diseases, including cancer, atherosclerosis, fibrosis, and multiple sclerosis [29–31]. Szasz et al. [32] have demonstrated that overexpression of SphK1 predicts poor overall survival [33]. However, the putative association between miR-124a and the Sphk1/S1P pathway needs to be comprehensively elucidated.

In the present study, we aimed to explore the clinical relevance of LINC00960 in LADC, as well as the targeted association between miR-124a and the Sphk1/S1P pathway. We hypothesized LINC00960 promoted the aggressiveness of lung adenocarcinoma via the miR-124a/SphK1 axis. Our findings may provide new evidence in terms of LADC prevention and therapy.

## Material and methods

### Clinical sample collection

A total of 60 clinical samples and 60 healthy subjects (half for male and half for female) were collected from patients with LADC, hospitalized at Jinan Central Hospital Affiliated to Shandong University. None of the patients underwent chemotherapy or radiotherapy prior to resection. The samples were immediately stored at −80°C after surgery. This study was approved by the Jinan Central Hospital Affiliated to Shandong University (no. SDU-20181219).

### Cell lines

The human bronchial epithelial cell line (BEAS-2B) and human LADC cell lines (PG49, H1299, PC-9 and A549) were purchased from CoBioer Biosciences Co., Ltd. Cells were cultured in RPMI-1640 medium containing 10% fetal bovine serum (FBS) and 1% penicillin/streptomycin at 37°C in 5% CO_2_.

### Cell transfection

LINC00960 overexpression plasmids, sh-LINC00960, mimic NC (the negative control), miR-124a mimic, inhibitor NC, miR-124a inhibitor, vector, or SphK1 were purchased from GenePharma, Shanghai. Transfection was performed using Lipofectamine® 2000 reagent.

### Quantitative reverse transcription-polymerase chain reaction (qRT-PCR)

Total RNA was isolated from cells, and cDNA was synthesized using a Reverse Transcription Kit. qPCR was subsequently performed using Power SYBR™ Green RNA-to-C_T_™ 1-Step Kit. The results were normalized to GAPDH and calculated using the 2^−ΔΔCT^ method [34]. The primer sequences are as follows:

LINC00960: Forward (5ʹ-3ʹ) CCTCTAAGCCTAAGCACCGCC; Reverse (5ʹ-3ʹ) GGAAGCCTGGGCAAGGAATGG.

miR-142a: Forward (5ʹ-3ʹ) GGTAAGGCACGCGGT; Reverse (5ʹ-3ʹ) CAGTGCGTGTCGTGGAGT.

Sphk1: Forward (5ʹ-3ʹ) AGCTTCCTTGAACCATTATGCTG; Reverse (5ʹ-3ʹ) AGGTCTTCATTGGTGACCTGCT.

GAPDH Forward (5ʹ-3ʹ) GGGAGCCAAAAGGGTCATCA; Reverse (5ʹ-3ʹ) TGATGGCATGGACTGTGGTC.

### Bioinformatic approaches

Possible targets of LINC00960 and miR-124a were predicted using online databases, DIANA and TargetScan.

### MTT assay

The cell viability was detected according to a previous study [35]. In brief, cells were trypsinized at a density of 1 × 104 cells/mL and the cell suspension was added to a 96-well plate (100 μL/well). Then, cells were cultured with 100 μL MTT solution. The supernatant was discarded, and 200 μL dimethyl sulfoxide solution (Macklin Biochemical Co., Ltd.) was added to each well. The solution was subsequently mixed well using a shaker; absorbance was measured at a wavelength of 490 nm using a microplate spectrophotometer.

### Transwell assay

The transwell assay was performed according to a previous research [36]. After transfection, cells were collected and seeded in the upper chamber, precoated with or without Matrigel matrix. Cells in the lower chamber were cultured with 600 μL DMEM containing 20% FBS. After 24 h of incubation at 37°C, the cells in the upper chamber were removed. The migrated or invaded cells were fixed and stained with 0.1% crystal violet. The number of migrated or invaded cells was counted using an inverted microscope.

### Colony-formation assay

As described by Lei et al. [37], cells were plated onto a 24-well plate. The cells were then cultured in RPMI-1640 medium for two weeks. Next, cells were fixed with 4% paraformaldehyde and stained with 0.1% crystal violet. Finally, the cells were visualized using an inverted light microscope.

### Luciferase reporter assays

The Luciferase reporter assay was carried out according to a previous study [38]. Wild-type (WT) and mutant (MUT) LINC00960 and SphK1 luciferase reporter vectors were constructed by RiboBio. Cells were co-transfected with WT/MUT vectors and mimic NC/miR −124a mimic (RiboBio Co., Ltd.) were co-transfected into A549 and H1299 cells. Then, cells were incubated for 24 h and lysed to detect luciferase activity using a dual-luciferase reporter gene assay kit (11402ES60; Yeasen Biotechnology (Shanghai) Co., Ltd.) 48 h after transfection.

### RNA pull-down assay

As decribed by Torres et al. [39]. The biotinylated miR-124a probe and control probe were synthesized by Shanghai Sangon Biology Engineering Technology Service, Ltd. The probe (50 pmol) was incubated with 50 μL Streptavidin-coated beads at 4°C for 2 h. Then, the cells were lysed to release total RNA, and the beads were subsequently washed six times in lysis buffer. After separation, the same qRT-PCR process described above was used to quantify the relative expression of SphK1.

### Western blotting

As described by Kurien et al. [40]. Total protein was collected from cells, and its concentration was measured using a BCA kit. The protein (60 μg) was then separated by 8% sodium dodecyl sulfate-polyacrylamide gel electrophoresis (SDS-PAGE) for 1.5 h at 90 V, followed by transfer of the separated proteins onto PVDF membranes for 2 h at 220 mA. Then, membranes were blocked using fat-free milk for 2 h, followed by incubation with primary and secondary antibodies. Finally, the results were captured using an enhanced chemiluminescence system.

### ELISA

The concentration of S1P in A549 cells was detected using an ELISA kit (ML-Elisa-0470; R&D Systems, Abnova), according to the manufacturer’s protocol. A549 cells were lysed and centrifuged at 10,000 rpm for 5 min, and the supernatant was collected.

### Establishment of xenograft tumor model using nude mice

Four-week-old female BALB/c nude mice (n = 20; Kay Biotech Co., Ltd.) were equally and randomly assigned to four groups: the antagomir control group, the antagomir-124a group, the agomir-control group, and the agomir-124a group. All mice were strictly bred under pathogen-free conditions with 12 h dark/light in separate cages and free access to food and water. Xenografts were induced by subcutaneously injecting A549 cells transfected with 50 nM antagomir-control, antagomir-124a, agomir-control, or agomir-124a, at a density of 2 × 106 cells/200 μL cell sap, into nude mice. The tumor volume was measured every three days (calculation method: V = ab^2^/2, where a is the long diameter and b is the short diameter). The maximum tumor diameter throughout the experimental course was measured as 12.4 mm. After 24 days, the mice were sacrificed.

### Immunohistochemical analysis

Xenograft tumors from the antagomir-control, antagomir-124a, agomir-control, and agomir-124a groups (see below) were resected and embedded in paraffin; xenograft tissues were sectioned into 4-μm-thick slices. After heating at 60°C in a thermotank for 120 min, the slices were dewaxed and rehydrated in grade ethanol. An H_2_O_2_ solution (3%) was then added. Subsequently, the slides were incubated in 0.01 M sodium citrate (pH 6.0) at 100°C for 20 min to expose the antigen. Next, the slices were washed with phosphate-buffered saline (PBS) and incubated with rabbit anti-human Ki67 antibody (AF7617; 1:200; R&D Systems, Inc.) at room temperature for 2 h. After washing the slides with PBS, the specimens were treated with a peroxidase reagent. After washing with PBS three times, an SP staining kit (Beijing Solarbio Science & Technology Co., Ltd.) was used for visualization. The Ki67-positive cells were counted under a light microscope by randomly selecting 10 viewing fields per filter.

### Statistical analysis

Data were analyzed using GraphPad 6.0 (GraphPad Software, Inc., La Jolla, CA, USA) and expressed as the mean ± standard deviation (SD). Differences were analyzed using Student’s t-test and ANOVA, followed by Duncan’s post hoc test. Differences were considered statistically significant at *P* < 0.05.

## Results

This study aimed to explore the role of LINC00960 in LADC. We demonstrated that LINC00960 was up-regulated in the LADC patients and cells, and promoting the growth and metastasis of LADC cells via miR-124a/SphK1 axis.

### LINC00960 was overexpressed in LADC

As shown in Figure 1a, the expression of LINC00960 in tumor tissues was significantly upregulated in the LADC patient compared with healthy persons (Figure 1a). Furthermore, LINC00960 was significantly upregulated in LADC cell lines (PG49, PC-9, A549, and H1299) when compared with the human bronchial epithelial cell line (BEAS- 2 B; Figure 1b).

**Figure 1.** LINC00960 is upregulated in LADC tissues and cells. (a) LINC00960 expression in clinical samples. (b) LINC00960 expression in LADC cells. **P < 0.01, vs. normal or BEAS-2B. LADC, lung adenocarcinoma.

### LINC00960 knockdown suppressed aggressiveness of A549 and H1299 cells

As shown in Figure 2a, the expression of LINC00960 was significantly increased by LINC00960 overexpression plasmids and decreased by sh-LINC00960, suggesting efficient transfection. Overexpression of LINC00960 significantly enhanced the viability of LADC cells, whereas LINC00960 knockdown suppressed the cell viability (Figure 2b). In addition, LINC00960 knockdown dramatically decreased the number of colonies, migrated and invaded cells, while overexpression of LINC00960 dramatically increased them. (Figure 2c-e).

**Figure 2.** LINC00960 overexpression suppresses the aggressiveness of LADC cells in vitro. (a) LINC00960 expression in LADC cells. (b) Cell viability of LADC cells. (c) Cell proliferation of LADC cells. (d) Migratory ability of LADC cells. (e) The invasion ability of LADC cells. **P < 0.01, *vs*. OE NC or sh-NC. LADC, lung adenocarcinoma. OE, over expression. NC, negative control. sh, short hairpin.

### LINC00960 knockdown suppressed the growth of LADC tumors in vivo

As shown in Figure 3a, the expression of *miR-124a* was significantly increased in the sh-LINC00960 group. Moreover, LINC00960 knockdown inhibited the LADC tumor growth, manifested as decreased tumor size, volume, and weight (Figure 3b and c). In the sh-LINC00960 group, resected xenograft tumors exhibited fewer Ki67-positive cells compared with the sh-NC group (Figure 3d).

**Figure 3.** LINC00960 can regulate the growth of LADC in vivo. (a) Relative expression of miR-124a in the agomir-124a group. (b and c) LINC00960 knockdown suppresses tumor growth. (d) Ki67-positive cells were imaged in xenograft slices. **P < 0.01, *vs*. sh-NC. LADC, lung adenocarcinoma. NC, negative control. sh, short hairpin.

### LINC00960 targeted miR-124a

To further investigate the potential of LINC00960 in LADC, we investigated the underlying mechanisms. The online database revealed binding sites between LINC00960 and miR-124a (Figure 4a). According to the luciferase assay results, miR-124a suppressed luciferase activity in the WT LINC00960 vector group of A5499 and H1299 cells, revealing that miR-124a could directly target the 3ʹ-untranslated region (3ʹ-UTR) of LINC00960 (Figure 4b). The RNA pull-down assay further confirmed the interaction between LINC00960 and miR-124a (Figure 4c). The expression of miR-124a was remarkably reduced in the LINC00960 OE group and increased in the sh-LINC00960 group (Figure 4d). Moreover, miR-124a was downregulated in LADC tissues and cells (Figure 4e and f).

**Figure 4.** LINC00960 targets miR-124a. (a) Binding sites between LINC00960 and miR-124a. (b) The interaction between LINC00960 and miR-124a was detected using a luciferase assay. (c) The interaction between LINC00960 and miR-124a was verified using the RNA pull-down assay. (d) Expression of miR-124a detected by qRT-PCR. (e) Expression of miR-124a in clinical samples. (f) Expression of miR-124a in LADC cells. **P < 0.01, *vs*. sh-NC. LADC, lung adenocarcinoma; qRT-PCR, quantitative reverse transcription-polymerase chain reaction. OE, over expression. NC, negative control. sh, short hairpin. WT, Wild-type. MUT, mutant-type.

Downregulated *miR-124a induced the aggressiveness of LADC cells*. miR-124a was significantly downregulated in the miR-124a inhibitor group (Figure 5a). Downregulation of miR-124a significantly increased the cell viability, number of colonies, migrated and invaded cells in the LADC cells compared with sh-LINC00960+ miR-124a inhibitor NC group. (Figure 5b-e).

**Figure 5.** Downregulated miR-124a promotes aggressiveness of LADC cells. (a) The transfection efficiency of miR-124a. (b) Cell viability of LADC cells. (c) Cell proliferation of LADC cells. (d) Migratory ability of LADC cells. (e) The invasion ability of LADC cells. **P < 0.01, *vs*. sh-NC, ^##^P < 0.01, vs. sh-LINC00960. LADC, lung adenocarcinoma. NC, negative control. sh, short hairpin.

### miR-124a directly targeted SphK1

Figure 6a presents the binding sites between miR-124a and SphK1. According to the luciferase assay results, miR-124a suppressed luciferase activity in the WT SphK1 vector group of A5499 and H1299 cells, revealing that miR-124a could directly target the 3ʹ-untranslated region (3ʹ-UTR) of SphK1 (Figure 6b). The RNA pull-down assay further confirmed the interaction between SphK1 and miR-124a (Figure 6c). LINC00960 knockdown significantly decreased the expression of SphK1, which was reversed by the miR-124a inhibitor (Figure 6d). Moreover, SphK1 secretion was remarkably upregulated in LADC tissues and cells (Figure 6e and f).

**Figure 6.** SphK1 is a target of miR-124a. (a) Binding sites between SphK1 and miR-124a. (b) miR-124a suppresses the luciferase activities controlled by SphK1 3ʹ‑UTR in A549 and H1299 cells. (c) Relative enrichment of SphK1 was analyzed by qRT-PCR. (d and e) SphK1 mRNA expression in clinical samples. (f) Relative mRNA expression of SphK1 in LADC cells. Three independent experiments were performed. **P < 0.01, *vs*. mimic NC or inhibitor NC. SphK1, sphingosine kinase 1; S1P, sphingosine-1-phosphate; LADC, lung adenocarcinoma; qRT-PCR, quantitative reverse transcription-polymerase chain reaction. NC, negative control. sh, short hairpin. WT, Wild-type. MUT, mutant-type.

### SphK1 promoted the aggressiveness of LADC cells

SphK1 was notably upregulated in the SphK1 OE group, suggesting successful transfection (Figure 7a). To better understand how the interaction between miR-124a and SphK1 influences LADC cell viability, proliferation, and migration, miR-124a and SphK1 were co-transfected into A549 and H1299 cells. SphK1 partially reversed the anti-tumor behaviors of miR-124a by increasing the proliferation, migration, and invasion abilities of LADC cells (Figure 7b-e).

**Figure 7.** Sphk1 reverses the inhibitory effects of miR-124a on cell viability, proliferation, and migration. (a) The SphK1 transfection efficiency. (b) Cell viability of LADC cells. (c) Cell proliferation of LADC cells. (d) Migratory ability of LADC cells. (e) The invasion ability of LADC cells. **P < 0.01, *vs*. mimic NC or miR-124a+vector. SphK1, sphingosine kinase 1; LADC, lung adenocarcinoma. NC, negative control.

## Discussion

In the present study, we investigated the role of LINC00960 in LADC. We observed that LINC00960 was overexpressed in LADC, whereas LINC00960 knockdown suppressed the proliferation, migration, and invasion of LADC cells by modulating the miR-124-3p/SphK1 axis.

In recent years, the potential of lncRNAs in cancer has gained momentum. In LADC, dysregulated lncRNAs, such as DGCR5, TTN-AS1, and GMDS-AS1, promote tumorigenesis [13–15]. Aberrant lncRNA expression has been associated with poor clinical outcomes. Therefore, these lncRNAs may function as tumor suppressors or oncogenes and may be therapeutic targets for LADC. LINC00960 acts as an oncogene in bladder cancer and pancreatic ductal adenocarcinoma, and its overexpression predicts poor clinical outcomes [16,17]. Herein, LINC00960 was overexpressed in LADC. However, its downregulation suppressed the aggressiveness of LADC cells, as well as tumor growth. Therefore, LINC00960 may function as an oncogene in LADC. Knockdown of LINC00960 may be an alternative to LADC treatment.

lncRNAs function as competing endogenous RNAs (ceRNAs) to participate in numerous biological processes by sponging miRNA(s) [10,15,17]. In the present study, miR-124a was a target miRNA for LINC00960. miRNAs are essential regulatory factors in the initiation and development of cancer [35]. Numerous studies have shown that miR-124a is aberrantly expressed in malignant tumors. For example, the expression of miR-124a is reportedly downregulated in acute lymphoblastic leukemia through hypermethylation of the promoter and via histone modifications [36]. miR-124a expression is downregulated in both uveal melanoma cells and tissues [37]. Moreover, miR-124a is shown to inhibit the progression of uveal melanoma both *in vivo* and *in vitro* [38]. Functionally, overexpression of miR-124a inhibits the progression of glioblastoma cells [39]. Luo et al. [26] have previously shown that miR-124a is a novel diagnostic and prognostic chemotherapeutic biomarker for NSCLC. These results implied that miR-124a might function as an anti-tumor miRNA in LADC. In the current study, miR-124a downregulated LADC, which is consistent with the findings of Luo et al. [26]. Furthermore, downregulation of miR-124a promoted the aggressiveness of LADC cells and tumor growth *in vitro*. Collectively, these findings suggest that LINC00960 may participate in the progression of LADC by sponging miR-124a. However, the underlying mechanism warrants further investigation.

Growing evidence has revealed that miRNAs participate in the progression of tumors by binding to the 3ʹUTR of their targets [22,27]. In the present study, SphK1 was predicted to be a target of miR-124a. SphK1 is an oncogenic enzyme in diverse cancers [40,41]. Notably, SphK1 promotes NSCLC development. Overexpression of SphK1 exacerbates the development of NSCLC by activating STAT3 [21,42–48]. Herein, LINC00960 sponged miR-124a to upregulate the expression of SphK1. Overexpression of SphK1 reversed the anti-tumor effects of miR-124a in LADC.

## Conclusion

In conclusion, LINC00960 was overexpressed in LADC. Conversely, downregulation of LINC00960 suppressed the aggressiveness of LADC by regulating the miR-124a/SphK1 axis. These findings provide novel insights into the function of LINC00960 in LADC.

## Highlights

1. LINC00960 sponged miR-124a to inhibit the SphK1/S1P pathway
2. LINC00960 knockdown suppressed the proliferation, migration, and invasion
3. LINC00960 may be a potential therapeutic biomarker for LADC
